The article "Manganese, Iron, Lead, and Zinc Levels and Haematological Profile among Welders in Bibiani Anhwiaso Bekwai District, Ghana" was published in 2022. Journal: J Environ Public Health.

# Manganese, Iron, Lead, and Zinc Levels and Haematological Profile among Welders in Bibiani Anhwiaso Bekwai District, Ghana

**DOI:** 10.1155/2022/1508523

**Published:** 2022-07-08

**Authors:** Isaac Bainin, Samuel Fosu Gyasi, Esi Awuah, Daniel Obeng-Ofori, Faisal Abdallah, Emmanuel Timmy Donkoh, Akwasi Asamoah, Robert Adu

**Affiliations:** ^1^Department of Civil & Environmental Engineering, The University of Energy and Natural Resources, Sunyani, Ghana; ^2^Department of Basic & Applied Biology, The University of Energy and Natural Resources, Sunyani, Ghana; ^3^Center for Research in Applied Biology, CeRAB, University of Energy and Natural Resources, Sunyani, Ghana; ^4^Department of Civil and Environmental Engineering, Kwame Nkrumah University of Science and Technology, Sunyani, Ghana; ^5^Office of the Vice-Chancellor, Catholic University, Fiapre, Ghana

## Abstract

Welders are exposed to metal ions or oxides through direct contact at occupational sites or indirectly through uptake from contaminated dust or air. This study was a case-control study designed to assess the levels of some heavy metals and the hematological profile of welders (cases) as compared to nonwelders (controls) from Bibiani Anhwiaso Bekwai District of Ghana, comparatively to determine whether their values are within acceptable international range. A quantitative-based survey using structured questionnaires was used to collect demographic data from purposively selected welders (*n* = 40) and nonwelders (*n* = 40) from the study area. Five (5 mL) blood samples were collected from the study participants and analyzed for blood cell count as well as levels of Mn, Fe, Pb, and Zn. There were no significant differences in the Mn, Zn, and Fe levels between the welders and nonwelders (*p*=0.431, 0.53 vs. 0.23 mg/L, *p*=0.05, 0.41 vs. 0.15, *p*=0.886, 1.82 vs. 1.11). The level of Pb was, however, significantly lower among welders compared to the nonwelders (*p*=0.016, 0.09 < 0.3 mg/L). The total white blood cell count did not differ significantly between welders and nonwelders (*p*=0.365, 5.16 vs. 4.85 × 10^9^/L). However, the mixed cell fraction was significantly higher among welders compared to nonwelders (*p*=0.027, 0.34 × 10^9^/L > 0.28* × *10^9^/L). Red blood cell count and indices showed no significant differences between the welders and nonwelders. Hemoglobin levels in welders were, however, higher (14.47 g/dL) but this was not statistically significant compared to their nonwelder counterparts (13.85 g/dL). It was concluded from the study that welders in Bibiani Anhwiaso Bekwai District of the Western Region of Ghana had elevated levels of Pb in their bodies. This was associated with an increase in mixed white blood cell fraction platelets. However, the recorded levels were within the accepted physiological limits suggesting that the heavy metal exposure of welders had no clinically pathological significance.

## 1. Introduction

Welding is one of the fundamental processes for joining pieces of metals together in the fabrication industry. Due to its relatively cheaper cost, it is a more preferred joining method compared to nailing, glue bonding, or riveting [1]. Different types of welding have been identified in commercial use, with electric arc welding being the most common. In electric arc welding, heat fusion (temperature above 4000°C) is produced when electricity passes through a gas between two electrical conductors [2]. When the electric welding arc is struck between electrode and base metal in the air or inert gas, the metal vapor, having evaporated at a very high temperature, is then cooled down in the gas stream and condenses to form fumes [3]. Although this practice generally is considered safe, welders are known to have an increased risk of mortality from fume-related lung disease, apart from lung cancer and pneumonia [4]. This is because inhalation of fumes from iron and steel causes benign and reversible pneumoconiosis known as siderosis [5].

During unprotected welding, there is generation of particulates and gases which can be inhaled and further leads to bioaccumulation [6]. The toxicity of welding fumes on the human body results from abnormal absorption, distribution, metabolism, and poor excretion of the main components of these fumes, such as heavy metals. Heavy metal is the generic term for metallic elements with an atomic weight higher than 40.04 [7]. This group includes Aluminium, Antimony, Arsenic, Beryllium, Cadmium, Chromium, Cobalt, Copper, Iron, Lead, Manganese, Molybdenum, Nickel, Silver, Tin, etc. [8]. These heavy metals, when present in welding fumes, can penetrate the human body through unprotected inhalation. Inside an organism, they bind to cellular structures, thereby damaging the performance of essential biological functions [9]. Heavy metals easily bind to the sulfhydryl groups of several enzymes that control the speed of metabolic reactions forming a metal-enzyme complex. These complexes lead to the loss of the catalytic activity of the enzyme over time with toxicity depending on factors including time of exposure, dose, and the health status of the people exposed (EEA, 2020).

The majority of these metals found in fumes can bioaccumulate in living systems during unprotected exposures [8]. The contamination chain of heavy metals almost always follows a cyclic order: industry, atmosphere, soil, water, food, and humans [10]. Toxicity and the resulting threat to human health of any contaminant are, of course, a function of concentration and it is well-known that chronic exposure to heavy metals and metalloids at relatively low levels can also cause adverse effects [11, 12].

Anemia and, less commonly, leukopenia, eosinophilia, thrombocytopenia, and pancytopenia have been reported due to heavy metal toxicity [13]. Most people exposed to heavy metals have normal red blood cell count; however, hematological effects were more, among nonoccupational settings [14]. The other two hematological effects reported due to heavy metal exposure include lymphocytosis and lymphopenia. Three studies ([14, 17]) reported a weak to moderate positive correlation between lymphocytes and mercury. One reported a mean difference [17] and the other two described an inverse association between lymphocytes and mercury exposure [15, 18]. These results confirm the relation or association between heavy metal exposure and hematological effects, especially for anemia, lymphopenia, lymphocytosis, neutrophilia, and basophilia. However, none of these studies could determine a causal relationship, as they were not designed for this purpose.

Bibiani Anhwiaso Bekwai District is a district in the rich mining area in the Western Region of Ghana. The district is predominantly made up of oxysterols soils, which are rich in mineral deposits making mining the most lucrative economic activity in the area. The most dominant mineral deposits are gold and bauxite. The companies dealing in these mining activities include Mesin Mensin Gold Limited at Bibiani; Chirano Goldfield Gold mines Limited at Chirano, and Bossai Bosai Minerals Limited at Awaso [19]. This has attracted many artisans, the majority of whom make a livelihood from welding. With the constant exposure to welding fumes from their daily operation, it is unclear whether their activity is impacting negatively on their health. To date, data on the toxicity level of this cadre of artisans is yet to be fully documented. This study sought to assess the levels of some heavy metals and the hematological profile of welders and nonwelders recruited from within the community.

## 2. Methodology

### 2.1. Study Design

A case-control study design was adopted for this study which commenced from September to October 2019.

### 2.2. Study Area

The Bibiani-Anhwiaso-Bekwai District was established in 1988 by Legislative Instrument (L.I) 1387 under the Local Government Law, 1988 (Provisional National Defence Council Law 207; PNDCL 207). The total land area of the district is 873 km square. The district attained municipal status in March 2018. The district is richly endowed with human and numerous natural resources, particularly natural tourist attraction sites. This ranges from a large number of labor, rich soil, minerals (Gold, Bauxite) good climatic conditions, tropical rainforest with a variety of timber species, cash crops, food crops, and livestock (GSS, 2010).

The district is bounded on the north by the Atwima Mponua District in the Ashanti Region; south by the Wassa Amenfi in the Western Region; west by the Sefwi Wiawso Municipality in the Western Region; east by the Denkyira North and Amansie East in the Central Region and Ashanti region, respectively (Figure 1).

### 2.3. Study Communities

The study was carried out in three (3) main communities in the district. The communities were Bibiani, Sefwi Bekwai, and Sefwi Tanoso.

### 2.4. Selection of Study Population

According to data from the Rural Technology Facility (RTF) of the Bibiani Anhwiaso Bekwai Municipal Assembly (BABMA), the municipality is estimated to have about 40 workshops that comprise both welding and other workshops on the same piece of land. The other artisans on the same premises with the welders are automechanics, sprayers, autoelectricians, etc. The number of artisans at these selected workshops is estimated to be 330. This is made up of one hundred and thirty (130) welders and two hundred (200) nonwelders.

### 2.5. Selection Criteria

To be included in the study, a participant had to be 15 years and above and should have spent more than 1 year working in their respective shops.

### 2.6. Sampling Size Estimation

Fifty (50) male welders were purposively recruited for the study. Fifty (50) nonwelders made up of forty-nine (49) males and one (1) female were also purposively recruited as a control for the study. The selection was based on the proximity of their workshops. Out of the one hundred (100) respondents, twelve (12) respondents were excluded from the study due to their high intake of alcohol which could affect the results. Eight (8) respondents, however, declined to participate in the human study. This brought a total of 80 subjects (40 welders and 40 nonwelders) who were recruited for blood sample collection. This followed a study conducted by [20] with slight modification.

### 2.7. Data Collection

A collection point was set up at the various locations from where all participants converged for blood sampling. With the help of a trained phlebotomist, about 5 mL of each of the respondents' blood samples was collected by venipuncture into EDTA (ethylenediamine tetraacetic acid) tubes and properly sealed. The tube was gently inverted 6–8 times to ensure proper mixing of the blood with the anticoagulant. The sample was placed upright in the tube rack within an ice chest, properly labeled, and transported to the laboratory.

### 2.8. Haematological Analysis

About 2 mL of each participant's samples with their sample identity (ID) and other relevant demographic information such as name, age, and sex were entered and saved on the Haematology Analyser (18-Parameter Haematology Analyser, ABX Micros ESV 60, Horiba, France, 2016) before analyses following the manufacturer's instructions. The sample tube was gently inverted 8 times and placed under the probe. Care was taken to ensure that the probe reached at least mid-depth into the sample. The results were displayed on the screen for review and validation.

### 2.9. Heavy Metals Analyses

Selected heavy metals assessed included Manganese (Mn), Iron (Fe), Zinc (Zn), and Lead (Pb) based on a study conducted by [21] with slight modification. About 3 mL of blood sample was collected from the median cubital vein in the arm were collected using disposable syringes. The samples were transferred to metal-free heparinized polypropylene vials. The collection tubes were labeled and transported on ice within 24 hours of sample collection. About 5 mL of HNO_3_ was added to 0.5 mL of blood sample in a 100 mL conical flask and left overnight. The resultant solution was digested on the hot plate. As the sample began to dry, a 5 mL mixture of concentrated HNO_3_ : HClO_4_ was added to the mixture at a ratio of 6 : 1. The digestion process was completed again on the hot plate. The resulting mixture was rinsed with 1% HNO_3,_ and the solution was topped up to 10 mL with distilled water. The resulting solutions were analyzed by Atomic Absorption Spectroscopy (AAS–Varian AA240FS) following the manufacturer's instruction [22]. The results were printed and stored in a laboratory results records book.

### 2.10. Measurement of Flow Rate

With the help of Scientific Kit Corporation air check MTX Sidekick sampling pump (224–52MTX Model) by filtration through Whatman membrane filters of a radius of 25 mm with a pore size of 3.0 *μ*m, the particulate matter (PM) samples from welding fumes were collected daily from 8 am to 4 pm for three days continuously (4th–6th September). The welding fumes were channeled into a flow rate detector with an embedded filter to extract the particles in the generated fumes. The high-volume sampler was operating at a flow rate of 2.2 L/min. Each sampling group was made of a filter holder manifold connected to the sampling pump by a Teflon tube. The particulates were collected on Whatman filter paper from the sampling point. The sampler was installed on top of a building approximately 4.0–6.0 m high above the ground level and separate from other buildings.

### 2.11. Weighing of Filter Papers

Filter papers used were placed in a desiccator for 24 hours and weighed before and after sampling. Mettler digital analytical balance with 0.01 mg readability was used. Each filter was weighed three times to obtain a constant and accurate weight before recording. Blank filter papers were also kept in a desiccator for 24 hours and weighed three times to obtain constant weight but were not exposed to air. They were kept in paper envelopes (for correction purposes). All filter handling was done using vinyl gloves to avoid contamination.

#### 2.11.1. Determination of Total Suspended Particulate (TSP) and Toxicity Potential (TP)

(1) $$\begin{array}{c} \text{Total Suspended Particulate}\left(\text{TSP}\right)=\frac{\left[\text{Final weight}\left(W_{j}\right)-\text{Initial weight}\left(W_{\left.j\right)}\right)\right]\times 10^{6}}{\text{Flow rate}\times \text{Sampling Period}}, \end{array}$$

*W*_*f*_ is the weight of filter paper after sampling in grams, *W*_*i*_ is the weight of filter paper before sampling in grams. The flow rate of welding fumes is (m^3^/min). Sampling period is in minutes (mins). 10^6^ = conversion from grams to micrograms.

Due to the daily exposure to PM, the probability of its effect on human health exists. Therefore, Toxicity Potentials (TPs) were calculated.

(2) $$\begin{array}{c} \text{Toxicity Potentials}\left(\text{TPs}\right)=\frac{\text{Mass concentration of the total suspended particulate}\left(\text{TSP}\right)}{\text{Limit for ambient particulate matter concertration}\left(230\mu g/m^{3}\right)}. \end{array}$$

### 2.12. Ethical Clearance

The study was approved with the issuance of an Ethical clearance certificate (CHRPE/AP/569/19) by the Committee on Human Research, Publication & Ethics, School of Medical Sciences/Komfo Anokye Teaching Hospital; College of Health Sciences, Kwame Nkrumah University of Science & Technology, Kumasi, Ghana. Written informed consent was obtained from each participant before involving them in the study.

### 2.13. Data Analysis

The data obtained were manually entered into Microsoft Excel software. Exploratory analyses were carried out to obtain descriptive statistics with the GraphPad Prism 6. Differences between proportions were tested using the Chi-square test at a significance value of *p* < 0.05. The use of the chi-square test was justified by the bivariate nature of the distributions between the various categorical variables of respondents and their profession (welders and nonwelders).

## 3. Results

Table 1 shows the demographic data of welders and nonwelders from Bibiani Anhwiaso Bekwai District. The modal age category was 21–25 years which was common for both groups. There were no significant differences between age categories (15–20, 21–25, 26–30, and 36–40) (*p* ≥ 0.05). The 31–35 age category for the welders (15%) compared to nonwelders (0%) was statistically significant (*p* ≤ 0.0011). The age category above 41 was more in the nonwelders (7%) than in their welding counterparts (1%) (*p* ≤ 0.0025). The greater majority of the welders (100%) and nonwelders (97.5%) were males. The majority of the welders (85%) and nonwelders (87.5%) were also Christians, as shown in Table 1.

Most of the nonwelders had attained education at least up to the secondary school level (72.5%). Most of the respondents from both categories were also single, i.e., welders (62.5%) and nonwelders (57.5%). Assessment of household size showed that welders (42.5%) had more than 7 people in their household compared to the nonwelders (40%), but this was not statistically significant. Comparatively, greater proportions of the respondents who were welders (50%) lived in rented houses compared to the nonwelders (55%), with few proportions of these perching with their friends (5%; welders and 5%; nonwelders), but these were not significant.

Table 2 shows some heavy metals profiles of welders and nonwelders within the study area. There were no significant differences in the Manganese, Zinc, and Iron levels between the welders and nonwelders (*p*=0.431, 0.53 vs. 0.23 mg/L, *p*=0.05, 0.41 vs. 0.15, *p*=0.886, 1.82 vs. 1.11). Additionally, the values fell below the WHO acceptable limits for bioaccumulation for the indicated metals. The level of Pb was, however, significantly lower among welders compared to the nonwelders (*p*=0.016, 0.09 < 0.3 mg/L), but this also fell within the World Health Organization (WHO) acceptable limit of the metal in living systems.

The hematological profile of welders and nonwelders in the study area is presented in Table 3. The total white blood cell count did not differ significantly between welders and nonwelders (*p*=0.365, 5.16 vs. 4.85 × 10^9^/L). The differential WBC count revealed that the lymphocyte and granulocyte fractions were comparable between the case and control groups. However, the mixed cell fraction was significantly higher among welders compared to nonwelders (*p*=0.027, 0.34 × 10^9^/L > 0.28* × *10^9^/L). Both levels, however, fell within the reference range (0.2–1.0 × 10^9^/L) as shown in Table 3. Percentage mixed cell fraction was also higher in welders compared to the nonwelders recruited for the study (*p*=0.006, 6.66 > 5.96%) (Table 3).

Red blood cell count showed no significant difference between the welders and nonwelders. The haemoglobin concentration and haematocrit levels in welders (14.47 g/dL, 37.47%) were higher than those of the nonwelders (13.85 g/dL, 36.47%), but these were not statistically significant (*p*=0.060, 0.358). There were no significant differences between the groups for all red blood cell indices, but the mean cell hemoglobin (MCH) and mean cell volume (MCV) were generally higher among the welders whilst the mean cell hemoglobin concentration (MCHC) was higher among the nonwelders. The red blood cell distribution width was comparable between the welders and nonwelders. The platelet count was significantly higher among welders (*p*=0.001, 265.2 > 227.0* × *10^9^/L). Assessment of plateletcrit also showed significantly higher levels in welders (0.33%) as against (0.29%) nonwelders (*p*=0.004). Despite the differences observed among the study group with some parameters, most of the results were within the normal reference range except for the plateletcrit.

The welding fumes were channeled into a flow rate detector with an embedded filter to extract the particles in the generated fumes. This was done for the 3 consecutive days and results showed that the 3^rd^ day's recording for particulate amounts in grams is the highest for all the 3 readings as presented in Table 4 and Figure 2. With the help of these measurements, the total suspended particulate (TSP) (149 *μ*g/m^3^) and the toxicity potential (TP) (0.65) were determined to help check whether they were within the accepted permissible limits of WHO (TSP = 230 *μ*g/m^3^, TP = 2.64–6.50). The TSP and TP were within the accepted WHO limits, but TSP was above the Ghana Standard Authority (GSA) permissible limits.*W*_*f*_ = 9.4 *W*_*i*_ = 1.44 Flow rate = 111 Sampling period = 8 hours (8 × 60 = 480 min).

(4) $$\begin{array}{c} \text{TSP}\left(\mu g/m^{3}\right)=\frac{\left(9.4-1.44\right)\times 10^{6}}{111\times 480}=149\left(\mu g/m^{3}\right),\\ \text{Toxicity Potentials}\left(\text{TPs}\right)=\frac{\text{Mass concentration of the suspended particulate}\left(\text{TSP}\right)}{\text{Limit for ambient particulate matter concentration}\left(230\mu g/m^{3}\right)},\\ \text{TP}=\frac{149\left(\mu g/m^{3}\right)}{230\left(\mu g/m^{3}\right)}=0.63. \end{array}$$

(3) $$\begin{array}{c} \text{Total Suspended Particulater}\left(\text{TSP}\right)=\frac{\left[\text{Final weight}\left(W_{f}\right)-\text{Initial weight}\left(W_{i}\right)\right]\times 10^{6}}{\text{Flow rate}\times \text{Sampling Period}}, \end{array}$$

## 4. Discussion

This is the first time the knowledge and adherence to occupational safety among welders and nonwelders have been investigated within the study area. The present study showed that age, gender, and educational background were key to one's choice of career. The majority of the respondents were males between 15 and 30 years, and the majority of them were educated up to the secondary school level. It has been reported in a study conducted on gender equality in education that a challenge for policymakers is that age, gender, and education played key roles in the choice of one's occupation [25]. A similar study carried out also showed that age, gender, and educational status were key determinants of one's choice of work [26]. The total white blood cell (WBC) count among welders was slightly higher among welders compared to nonwelders (5.16 > 4.85, *p*=0.365) although this was not statistically significant, and both were within the normal reference ranges. Among the WBC differentials, only the monocyte fraction demonstrated significant variation between the two groups being compared, with welders having a slightly raised absolute count (0.34 > 0.28 (×10^9^/L), *p*=0.027) and a fraction (6.66 > 5.96%, *p*=0.006). Here, the response of phagocytes in inflammatory conditions as a result of foreign particles is the plausible explanation for the increased monocyte count and fraction among welders as compared to nonwelders. Reference [27] revealed in a study to investigate the systemic inflammatory responses following welding inhalation challenge test in a given population that number of leukocytes and neutrophils increased significantly following mild steel and stainless-steel welding challenge tests. This was also seen in a related study assessing the effects of welding fumes on hematological parameters of male albino rats (*Rattus norvegicus*). The study further related cute systemic inflammatory response to welding fume exposure and this showed a similar response for WBC count [28].

The red blood cell count and other RBC indices showed no significant difference between welders and nonwelders. All red blood cell (RBC) parameters were within the normal reference ranges for both cases and controls [29, 30]. In contrast to the findings of this study, [31] reported in their study in the Radiology department of Khuzestan province in Iran that the RBC count obtained for the workers from the exposed group was below that of the control. Reduced red blood cell production was not replicated in our case group because most of the heavy metals assessed had similar levels in both groups except for lead (Pb), for which the difference between the cases had lower levels.

In another study, the hemoglobin concentration determined for the workers was higher than that of the control, which was a result of cement dust [32]. Though no differences were identified in the hematocrit (HCT) values of the groups in this study, in previous research conducted in India among petrol pump workers, the mean HCT value for the workers was higher than the control. The difference was associated with exposure to air pollutants such as carbon monoxide (CO) in the workplace [33].

The platelet count was significantly higher in welders (265.2 > 227.0* *×* *10^9^/L, *p* < 0.01) though they were both within the normal reference range. The plateletcrit (PCT) was elevated in the case group as compared to the control group (0.33 > 0.29, *p* < 0.01). It follows that an increased platelet count would cause the platelet fraction of the blood to increase.

Reference [34] reported on hematological analysis in biomedical and pharmacological studies, where the PCT levels in the blood sample for the cases were a bit higher than the control, and this was in line with the current study.

The amount of total suspended particulate (TSP) obtained from the current study was less than the WHO's recommended guideline values [35, 36]. This also meant that although many welders generated a huge amount of welding fumes with particulates, it was not enough to cause harm to the welders. Workers at the workshop were found to be far less at risk in terms of toxicity potential (TP). Previous studies have revealed that it was only unprotected artisans who were constantly exposed to more than the WHO levels of TSP that were likely to be injured [37].

Hematological parameters such as RBC count, hematocrit value, and Hb profile are sensitive indicators of heavy metal stress on metabolism [38]. In the present study, although heavy metal levels were comparable between the two groups, the consistent rise or fall in the complete blood count parameters for the welders, though not significant, suggests some level of effect on these welders, which may be present in a larger sample size. Heavy metals act directly on hematopoietic stem cells in the bone marrow, causing a mechanical failure of the stem cells, impeding RBC production, and inducing carcinogenic changes in the WBC precursors [39].

Toxic manifestations of metals range from minor upper respiratory irritation, flu, cough, rhinitis, and nasal allergy to asthmatic attacks, chronic bronchitis, congestive chest diseases, high incidence of chronic obstructive pulmonary diseases (COPDs), and even lung cancer [40]. Heavy metal toxicity is a major environment-related health hazard to the populace and a risk factor for both acute and chronic respiratory illnesses. Even very low concentrations of heavy metals are sufficient to adversely affect the respiratory tract [41].

## 5. Conclusions

It was concluded from the study that welders in Bibiani Anhwiaso Bekwai District of the Western Region of Ghana had elevated levels of Mn and Fe in their bodies, with males between 31 and 35 years being the worst affected. This was associated with an increase in mean cell fraction, mean cell fraction percentage, platelets, and platelet numbers in these groups of artisans. This could be attributed to the noncompliance to using the appropriate personal protective equipment. The total suspended particulate and the toxicity potential were, however, low, falling within the acceptable limits of the World Health Organization [36]. This has future public health implications for this group of artisans if the situation is left unchecked. It is therefore recommended that education be intensified to enlighten the welders in the study area about the dangers of not donning the right personal protective equipment during welding.

## Figures and Tables

**Figure 1:** Study area of Bibiani Anhwiaso Bekwai Municipality.

**Figure 2:** Measurement of the flow rate of welding fumes and filter paper (a graphical representation of Table 4).

**Table 1:** Demography of study population stratified by welders and nonwelders (type of work).

Variable	Total (%)	Welders (%)	Non-welders (%)	*p* value	OR
Gender					
Male	79 (98.75)	40 (100)	39 (97.5)	0.314	3.08
Female	1 (1.25)	0 (0)	1 (2.5)	0.314	0.33

Age					
41 plus	8 (10.00)	1 (2.5)	7 (17.5)	0.025	0.12
36–40	9 (11.25)	5 (12.5)	4 (10.0)	0.724	1.29
31–35	6 (7.50)	6 (15.0)	0 (0.0)	0.011	15.26
26–30	8 (10.00)	3 (7.5)	5 (12.5)	0.456	0.57
21–25	29 (36.25)	16 (40.0)	13 (13.5)	0.485	1.39
15–20	20 (25.00)	9 (22.5)	11 (27.5)	0.606	0.77

Religion					
Islam	10 (12.50)	6 (15.0)	4 (10.0)	0.499	1.59
Christianity	69 (86.25)	34 (85.0)	35 (87.5)	0.745	0.81
Atheist	1 (1.25)	0 (0.0)	1 (2.5)	0.314	0.33

Educational status					
Basic	6 (7.50)	4 (10.0)	2 (5.0)	0.400	2.11
Secondary	56 (70.00)	27 (67.5)	29 (72.5)	0.626	0.79
Post sec	17 (21.25)	9 (22.5)	8 (20.0)	0.785	1.61
Tertiary	1 (1.25)	0 (0.0)	1 (2.5)		

Marital status					
Single	48 (60.00)	25 (62.5)	23 (57.5)	0.642	1.23
Married	32 (40.00)	15 (37.5)	17 (42.5)	0.648	0.81

Household size					
1 to 2	17 (21.25)	7 (17.5)	10 (25.0)	0.412	0.64
3 to 4	18 (22.50)	10 (25.0)	8 (20.0)	0.592	1.33
5 to 6	12 (15.00)	6 (15.0)	6 (15.0)	1.000	1.00
7 and above	33 (41.25)	17 (42.5)	16 (40.0)	0.820	1.11

Number of dependants					
1 to 2	36 (45.00)	16 (40.0)	20 (50.0)	0.369	0.67
3 to 4	16 (20.00)	8 (20.0)	8 (8.0)	1.000	1.00
5 to 6	11 (13.75)	3 (7.5)	8 (20.0)	0.105	0.32
7 and above	7 (8.75)	3 (7.5)	4 (10.0)	0.692	0.73

Housing					
Family house	20 (25.00)	10 (25.0)	10 (25.0)	1.000	1.00
Rented	42 (52.50)	20 (50.0)	22 (55.0)	0.654	0.82
Owned	14 (17.50)	8 (20.0)	6 (15.0)	0.556	1.42
Perching	4 (5.00)	2 (5.0)	2 (5.0)	1.000	1.00

*p* value: univariate *p* value; ^#^*p* value: multivariate *p* value; OR: odds ratio.

**Table 2:** Heavy metals profile of welders compared to the control.

Parameter	Heavy metals		WHO reference range	*p* value
	Non-welders (control)	Welders		
Mn (mg/L)	0.23	0.53	16–26 mg/L	0.431
Pb (mg/L)	0.3	0.09	0.99 mg/L	0.016
Zn (mg/L)	0.15	0.41	800–1200 mg/L	0.050
Fe (mg/L)	1.11	1.82	(6–200) × 10^−6^ mg/L	0.886

[23].

**Table 3:** Hematological parameters analysis of participants in the study area.

Parameter	FBC (S.E.M)		Reference ranges	*p* value
	Nonwelders (control)	Welders		
WBC (×109/L)	4.85	5.16	3.4–9.2	0.365
LYM (×109/L)	1.55	1.72	1.2–4.4	0.192
MON (×109/L)	0.28	0.34	0.2–1.0	**0.027**
GRAGRA (×109/L)	3.08	2.93	1.5–5.6	0.585
LYM (%)	31.40	34.24	25.2–57.7	0.090
MON (%)	5.96	6.66	5.3–16.3	**0.006**
GRA (%)	62.64	59.94	32.0–68.1	0.170
RBC (×1012/L)	5.67	4.99	3.4–5.8	0.381
HGB (g/L)	13.85	14.49	9.8–16.0	0.060
HCT (%)	36.47	37.47	28.9–48.7	0.358
MCV (fL)	75.23	75.57	72–97	0.841
MCH (pg)	28.72	29.23	22.6–33.5	0.384
MCHC (g/dL)	38.14	38.07	30.5–36.2	0.818
RDW-SD (%)	50.83	50.03	11.5–16.7	0.231
PLT (×109/L)	227.00	265.20	89–380	**0.001**
MPV (fL)	13.13	13.01	7.5–13.5	0.431
PDW (%)	17.06	17.40	12.6–23.0	0.504
PCT (%)	0.29	0.33	0.2–0.25	**0.004**

WBC: total white blood cell count, LYM (×10^9^/L): lymphocyte count, MON (×10^9^/L): monocyte count, GRA (×10^9^/L): granulocyte count, LYM (%): lymphocyte fraction, MONO (%): monocyte fraction, GRA (%): Granulocyte fraction, RBC: red blood cell count, HGB: hemoglobin concentration, HCT: hematocrit, MCV: mean cell volume, MCH: mean cell hemoglobin, MCHC: mean cell hemoglobin concentration, RDW-SD: red cell distribution width-standard deviation, PLT: platelet count, MPV: mean platelet volume, PDW: platelet distribution width, PCT: plateletcrit; Reference ranges obtained from [25] [24]

**Table 4:** measurement of flow rate of welding fumes and filter paper.

Readings/days	Initial (g) (00 hour)	Final (g) (after 8 hours)	Flow rate (m^3^/min)
1	1.42	8.40	112
2	1.42	9.70	120
3	1.47	10.10	100
Average	1.44	9.40	111

## Data Availability

The data for this work are available upon request.
